# Artificial blood

**DOI:** 10.4103/0972-5229.43685

**Published:** 2008

**Authors:** Suman Sarkar

**Affiliations:** **From:** Department of Anesthesiology, IMS Banaras Hindu University, Varanasi-221 105, Uttar Pradesh, India

**Keywords:** Blood, artificial blood, Perfluorocarbons

## Abstract

Artificial blood is a product made to act as a substitute for red blood cells. While true blood serves many different functions, artificial blood is designed for the sole purpose of transporting oxygen and carbon dioxide throughout the body. Depending on the type of artificial blood, it can be produced in different ways using synthetic production, chemical isolation, or recombinant biochemical technology. Development of the first blood substitutes dates back to the early 1600s, and the search for the ideal blood substitute continues. Various manufacturers have products in clinical trials; however, no truly safe and effective artificial blood product is currently marketed. It is anticipated that when an artificial blood product is available, it will have annual sales of over $7.6 billion in the United States alone.

## Background

Blood is a special type of connective tissue that is composed of white cells, red cells, platelets, and plasma. It has a variety of functions in the body. Plasma is the extracellular material made up of water, salts, and various proteins that, along with platelets, encourages blood to clot. Proteins in the plasma react with air and harden to prevent further bleeding. The white blood cells are responsible for the immune defense. They seek out invading organisms or materials and minimize their effect in the body.

The red cells in blood create the bright red color. As little as two drops of blood contains about one billion red blood cells. These cells are responsible for the transportation of oxygen and carbon dioxide throughout the body. They are also responsible for the “typing” phenomena. On the membranes of these cells are proteins that the body recognizes as its own. For this reason, a person can use only blood that is compatible with her type. Currently, artificial blood products are only designed to replace the function of red blood cells. It might even be better to call the products being developed now, oxygen carriers instead of artificial blood.

## History

There has been a need for blood replacements for as long as patients have been bleeding to death because of a serious injury. According to medical folklore, the ancient Incas were responsible for the first recorded blood transfusions. No real progress was made in the development of a blood substitute until 1616, when William Harvey described how blood is circulated throughout the body. In the years to follow, medical practitioners tried numerous substances such as beer, urine, milk, plant resins, and sheep blood as a substitute for blood. They had hoped that changing a person's blood could have different beneficial effects such as curing diseases or even changing a personality. The first successful human blood transfusions were done in 1667. Unfortunately, the practice was halted because patients who received subsequent transfusions died.

Of the different materials that were tried as blood substitutes over the years, only a few met with minimal success. Milk was one of the first of these materials. In 1854, patients were injected with milk to treat Asiatic cholera. Physicians believed that the milk helped regenerate white blood cells. In fact, enough of the patients given milk as a blood substitute seemed to improve that it was concluded to be a safe and legitimate blood replacement procedure. However, many practitioners remained skeptical so milk injections never found widespread appeal. It was soon discarded and forgotten as a blood replacement.

Another potential substitute was salt or saline solutions. In experiments done on frogs, scientists found that they could keep frogs alive for some time if they removed all their blood and replaced it with a saline solution. These results were a little misleading, however, because it was later determined that frogs could survive for a short time without any blood circulation at all. After much research, saline was developed as a plasma volume expander.

Other materials that were tried during the 1800s include hemoglobin and animal plasma. In 1868, researchers found that solutions containing hemoglobin isolated from red blood cells could be used as blood replacements. In 1871, they also examined the use of animal plasma and blood as a substitute for human blood. Both of these approaches were hampered by significant technological problems. First, scientists found it difficult to isolate a large volume of hemoglobin. Second, animal products contained many materials that were toxic to humans. Removing these toxins was a challenge during the nineteenth century.

A significant breakthrough in the development of artificial blood came in 1883 with the creation of Ringer's solution—a solution composed of sodium, potassium, and calcium salts. In research using part of a frog's heart, scientists found that the heart could be kept beating by applying the solution. This eventually led to findings that the reduction in blood pressure caused by a loss of blood volume could be restored by using Ringer's solution. This product evolved into a human product when lactate was added. While it is still used today as a blood-volume expander, Ringer's solution does not replace the action of red blood cells so it is not a true blood substitute.

Karl Landsteiner [Figure 1], who has been called the father of immunology, was the only child of Leopold Landsteiner, a prominent Austrian journalist and editor, and Fanny Hess Landsteiner. Landsteiner was educated at the University of Vienna, where he received his medical degree in 1891. While in medical school, Landsteiner began experimental work in chemistry, as he was greatly inspired by Ernst Ludwig, one of his professors. After receiving his medical degree, Landsteiner spent the next five years doing advanced research in organic chemistry for Emil Fischer, although medicine remained his chief interest. During 1886-1897, he combined these interests at the Institute of Hygiene at the University of Vienna where he researched immunology and serology. Immunology and serology then became Landsteiner's lifelong focus. Landsteiner was primarily interested in the lack of safety and effectiveness of blood transfusions. Prior to his work, blood transfusions were dangerous and underutilized because the donor's blood frequently clotted in the patient. Landsteiner was intrigued by the fact that when blood from different subjects was mixed, the blood did not always clot. He believed there were intrinsic biochemical similarities and dissimilarities in blood.

**Figure 1:** Karl Landsteiner

Using blood samples from his colleagues, he separated the blood's cells from its serum, and suspended the red blood cells in a saline solution. He then mixed each individual's serum with a sample from every cell suspension. Clotting occurred in some cares; in others there was no clotting. Landsteiner determined that human beings could be separated into blood groups according to the capacity of their red cells to clot in the presence of different serums. He named his blood classification groups A, B, and O. A fourth group AB, was discovered the following year. The result of this work was that patient and donor could be blood-typed beforehand, making blood transfusion a safe and routine medical practice. This discovery ultimately earned Landsteiner the 1930 Nobel Prize in physiology or medicine.

Blood transfusion research did not move forward until scientists developed a better understanding of the role of blood and the issues surrounding its function in the body. During World War I, a gum-saline solution containing galactoso-gluconic acid was used to extend plasma. If the concentration, pH, and temperature were adjusted, this material could be designed to match the viscosity of whole blood, allowing physicians to use less plasma. In the 1920s, studies suggested that this gum solution had some negative health effects. By the 1930s, the use of this material had significantly diminished. World War II reignited an interest in the research of blood and blood substitutes. Plasma donated from humans was commonly used to replace blood and to save soldiers from hemorrhagic shock. Eventually, this led to the establishment of blood banks by the American Red Cross in 1947.

In 1966, experiments with mice suggested a new type of blood substitute, perfluorochemicals (PFC). These are long chain polymers similar to Teflon. It was found that mice could survive even after being immersed in PFC. This gave scientists the idea to use PFC as a blood thinner. In 1968, the idea was tested on rats. The rat's blood was completely removed and replaced with a PFC emulsion. The animals lived for a few hours and recovered fully after their blood was replaced.

However, the established blood bank system in developed countries worked so well that research on blood substitutes waned in those countries. It received renewed interest when the shortcomings of the blood bank system were discovered during the Vietnam conflict. This prompted some researchers to begin looking for hemoglobin solutions and other synthetic oxygen carriers. Research in this area was further fueled in 1986 when it was discovered that HIV and hepatitis could be transmitted via blood transfusions.

## Design

The ideal artificial blood product has the following characteristics. First, it must be safe to use and compatible within the human body. This means that different blood types should not matter when an artificial blood is used. It also means that artificial blood can be processed to remove all disease-causing agents such as viruses and microorganisms. Second, it must be able to transport oxygen throughout the body and release it where it is needed. Third, it must be shelf stable. Unlike donated blood, artificial blood can be stored for over a year or more. This is in contrast to natural blood which can only be stored for one month before it breaks down. There are two significantly different products that are under development as blood substitutes. They differ primarily in the way that they carry oxygen. One is based on PFC, while the other is a hemoglobin-based product.

### Perfluorocarbons (PFC)

As suggested, PFC are biologically inert materials that can dissolve about 50 times more oxygen than blood plasma. They are relatively inexpensive to produce and can be made devoid of any biological materials. This eliminates the real possibility of spreading an infectious disease via a blood transfusion. From a technological standpoint, they have two significant hurdles to overcome before they can be utilized as artificial blood. First, they are not soluble in water, which means to get them to work they must be combined with emulsifiers—fatty compounds called lipids that are able to suspend tiny particles of perfluorochemicals in the blood. Second, they have the ability to carry much less oxygen than hemoglobin-based products. This means that significantly more PFC must be used. One product of this type has been approved for use by the Federal Drug Administration (FDA), but it has not been commercially successful because the amount needed to provide a benefit is too high. Improved PFC emulsions are being developed but have yet to reach the market.

### Hemoglobin-based products

Hemoglobin carries oxygen from the lungs to the other tissues in the body. Artificial blood based on hemoglobin takes advantage of this natural function. Unlike PFC products where dissolving is the key mechanism, oxygen covalently bonds to hemoglobin. These hemoglobin products are different than whole blood in that they are not contained in a membrane so the problem of blood typing is eliminated. However, raw hemoglobin cannot be used because it would break down into smaller, toxic compounds within the body. There are also problems with the stability of hemoglobin in a solution. The challenge in creating a hemoglobin-based artificial blood is to modify the hemoglobin molecule so these problems are resolved. Various strategies are employed to stabilize hemoglobin. This involves either chemically cross-linking molecules or using recombinant DNA technology to produce modified proteins. Just as Polyethylene Glycol-Modified Liposome-Encapsulated Hemoglobin, nanoparticle and polymersome encapsulated hemoglobin, stabilized hemoglobin solutions, polymerized hemoglobin solutions, conjugated hemoglobin solutions.

**Figure:** Artificial blood can be produced in different ways using synthetic production, chemical isolation, or recombinant biochemical technology. Synthetic hemoglobin-based products are produced from hemoglobin harvested from an E. coli bacteria strain. The hemoglobin is grown in a seed tank and then fermented

Conjugation of hemoglobin effectively increases its molecular size and reduces antigenicity, resulting in a slow rate of removal from the circulation and reduced “visibility” to the reticuloendothelial system. Unique features of conjugated hemoglobins are their high oncotic pressure, which makes them very potent plasma-volume expanders, and their viscosity.

Intramolecular cross-linked hemoglobins are not significantly increased in molecular weight but have specific chemical cross-links between polypeptide chains that prevent dissociation to dimers or monomers.

These modified hemoglobins are stable and soluble in solutions. Theoretically, these modifications should result in products that have a greater ability to carry oxygen than our own red blood cells. It is anticipated that the first of these products will be available within one to two years.

## Raw Materials

Depending on the type of artificial blood that is made, various raw materials are used. Hemoglobin-based products can use either isolated hemoglobin or synthetically produced hemoglobin.

To produce hemoglobin synthetically, manufacturers use compounds known as amino acids. These are chemicals that plants and animals use to create the proteins that are essential for life. There are 20 naturally occurring amino acids that may be used to produce hemoglobin. All of the amino acid molecules share certain chemical characteristics. They are made up of an amino group, a carboxyl group, and a side chain. The nature of the side chain differentiates the various amino acids. Hemoglobin synthesis also requires a specific type of bacteria and all of the materials needed to incubate it. This includes warm water, molasses, glucose, acetic acid, alcohols, urea, and liquid ammonia.

For other types of hemoglobin-based artificial blood products, the hemoglobin is isolated from human blood. It is typically obtained from donated blood that has expired before it is used. Other sources of hemoglobin come from spent animal blood. This hemoglobin is slightly different from human hemoglobin and must be modified before being used.

## The Manufacturing Process

The production of artificial blood can be done in a variety of ways. For hemoglobin-based products, this involves isolation or synthesization of hemoglobin, molecular modification then reconstitution in an artificial blood formula. PFC products involve a polymerization reaction. A method for the production of a synthetic hemoglobin-based product is outlined below.

### Hemoglobin synthesis

- To obtain hemoglobin, a strain of *E. coli* bacteria that has the ability to produce human hemoglobin is used. Over the course of about three days, the protein is harvested and the bacteria are destroyed. To start the fermentation process, a sample of the pure bacteria culture is transferred to a test tube that contains all the nutrients necessary for growth. This initial inoculation causes the bacteria to multiply. When the population is great enough, they are transferred to a seed tank.
- A seed tank is a large stainless steel kettle that provides an ideal environment for growing bacteria. It is filled with warm water, food, and an ammonia source which are all required for the production of hemoglobin. Other growth factors such as vitamins, amino acids, and minor nutrients are also added. The bacterial solution inside the seed tank is constantly bathed with compressed air and mixed to keep it moving. When enough time has passed, the contents of the seed tank is pumped to the fermentation tank.
- The fermentation tank is a larger version of the seed tank. It is also filled with a growth media needed for the bacteria to grow and produce hemoglobin. Since pH control is vital for optimal growth, ammonia water is added to the tank as necessary. When enough hemoglobin has been produced, the tank is emptied so isolation can begin.
- Isolation begins with a centrifugal separator that isolates much of the hemoglobin. It can be further segregated and purified using fractional distillation. This standard column separation met hod is based on the principle of boiling a liquid to separate one or more components and utilizes vertical structures called fractionating columns. From this column, the hemoglobin is transferred to a final processing tank.

### Final processing

- Here, it is mixed with water and other electrolytes [Figure 2] to produce the artificial blood. The artificial blood can then be pasteurized and put into an appropriate packaging. The quality of compounds is checked regularly during the entire process. Particularly important are frequent checks made on the bacterial culture. Also, various physical and chemical properties of the finished product are checked such as pH, melting point, moisture content, etc. This method of production has been shown to be able to produce batches as large as 2,640 gal (10,000 L).

**Figure 2:** Once fermented, the hemoglobin is purified and then mixed with water and other electrolytes to create useable artificial blood

## The Future

Currently, there are several companies working on the production of a safe and effective artificial blood substitute. The various blood substitutes all suffer from certain limitations. For example, most of the hemoglobin-based products last no more than 20-30h in the body. This compares to transfusions of whole blood that lasts 34 days. Also, these blood substitutes do not mimic the blood's ability to fight diseases and clot. Consequently, the current artificial blood technology will be limited to short-term blood replacement applications. In the future, it is anticipated that new materials to carry oxygen in the body will be found. Additionally, longer lasting products should be developed, as well as products that perform the other functions of blood.

